The article "The Comparative Pharmaco- and Histokinetics of the Therapeutic Dose of Estradiol Valerate and Bromocriptine in Common Quails" was retracted in 2024. Reasons: signs of a paper mill; suspected computer-generated content; unreliable results or conclusions; concerns about the data.

# The Comparative Pharmaco- and Histokinetics of the Therapeutic Dose of Estradiol Valerate and Bromocriptine in Common Quails

**DOI:** 10.1155/2022/5482895

**Published:** 2022-10-11

**Authors:** Muhammad Nadeem, Mehr-un Nisa, Maria Hussain Bangash, Zain Ul Abideen, Rukhsana Sattar, Huma Sattar, Muhammad Saif Ullah, Tahira Ruby, Aleem Ahmed Khan, Aqeel Ahmad

**Affiliations:** ^1^Department of Zoology, Ghazi University, Dera Ghazi Khan, Pakistan; ^2^Basic Health Unit, Khuda Bakhsh Mahar District Bahawalpur, Pakistan; ^3^Basic Health Unit 14/8R, Khanewal, Pakistan; ^4^Department of Biotechnology, The University of Lahore, Pakistan; ^5^Department of Zoology, Bahauddin Zakariya University, Multan, Pakistan; ^6^University of Chinese Academy of Science (UCAS), Beijing, China

## Abstract

The current study is aimed at examining the overall effects of steroids on the tissues of organisms and pharmacotherapeutics and pharmaco-histokinetics of several steroids, including Bromocriptine as mesylate and estradiol valerate in common quails (*Coturnix coturnix*). A total of 100 birds were used for pharmaco-histokinetics. The research was carried out in two separate trials, one during the fall season and the other during the spring season. Each experiment lasted for five, ten, fifteen, and twenty days. Each study group used 20 birds while basing their experiments on a control group of 5. At the stretch of five, ten, fifteen, and twenty days in each season, therapeutic dosages were administered to a sum of two groups representing two separate steroid trial groups. Each steroid was administered to each bird in a therapeutic dose, which was three drops administered twice daily. Clinical symptoms include despondency, sluggishness, and variations in weight and temperature that almost all treated birds display. However, only in trials conducted in the fall was a sizable degree of body enlargement in one treated bird noticed. The winter testing showed a mortality rate. Four birds have died in the twenty-day group. One bird died when treated with estradiol valerate, and three birds died treated with Bromocriptine as mesylate. Both the male and female birds showed signs of having lost some of their body weight. The treated birds' kidney, stomach, hearts, and livers exhibited some edema. In comparison, almost all birds show enteritis, which indicates that steroids mainly affect the intestine. There were apparent differences in the histological analysis of heart and skeletal muscle and some treated birds with the control group. The kidney, liver, and intestine show the major histopathological change in all treated birds.

## 1. Introduction

All the steroids are synthesised from the lanosterol in the cell. Lanosterol is the naturally occurring compound found in animals, plants, fungi, and some bacteria. The synthesis of steroids is called steroidogenesis [1]. The release of steroids and their mechanism of action are regulated by neuronal and hormonal signals. The pituitary gland is stimulated by neural impulses from the hypothalamus; the pituitary gland then releases a hormone that influences the ovaries, kidneys, and testicles to regulate hormonal levels through a feedback process [1, 2]. The first steps of steroid production are performed in mitochondria. Cholesterol is converted to pregnenolone in mitochondria by the enzyme p450sec [3]. The current study reveals that steroid output is controlled by steroid metabolism, i.e., biosynthesis. In order to protect the cellular membranes against antifungal medications like amphotericin B and azol, fungus synthesise ergosterols [4]. In female humans and other animals, steroids increase sickness and the immune system's reaction [5]. Numerous physiological processes in vertebrates, including responsiveness and electrolyte balance, are influenced by corticosteroids [6]. Canada, Europe, US, and other countries throughout the world all utilise estradiol valerate. Estradiol valerate has been used by women to prevent pregnancy for more than 50 years. [7]. Estradiol valerate is a hormone that is utilised in the treatment of a variety of conditions, including transgender women, menopausal symptoms, low oestrogen levels, and hormonal birth control [8]. Estradiol valerate at large doses raises the risk of thrombosis, alters the lipid profile in the blood, and raises the level of both prolactin and insulin resistance [9]. The Control Centers for Disease claim that, between 2006 and 2008, 10.5 million persons used oral contraceptives containing estradiol valerate as a birth control method [10]. When testosterone is given to a female, the female is unable to reproduce and has fewer cloacal glands. In fact, estradiol-17 is applied to male quail to promote copulation and 5-dihydrotestosterone to promote cloacal gland development [11].

The article "The Comparative Pharmaco- and Histokinetics of the Therapeutic Dose of Estradiol Valerate and Bromocriptine in Common Quails" was retracted in 2024. Reasons: signs of a paper mill; suspected computer-generated content; unreliable results or conclusions; concerns about the data.

By inhibiting ovulation and using its hormone, estradiol valerate prevents conception. The endometrium and cervical mucus have changed, making it difficult for sperm to penetrate. Bromocriptine use over an extended period of time results in anxiety, agitation, suicidal thoughts, weariness, and irritability [12]. Gallstone formation and cholesterol retention are more likely to occur when the gallbladder is not completely empty in late pregnancy. Gallstone development and cholesterol retention are both increased during pregnancy [13]. During the neonatal stage and during social interactions, steroids have an impact on a mammal's body [13].

The social behaviors of mammals can be modified by altering the hormone concentration (neuropeptides) [14]. They affect the human body in a number of ways. The primary impacts on the body alter mood and raise the dangers of anxiety, sadness, and menopause [15]. The birds' immunological function is inhibited by stress, their immunity is decreased, and pathogens can easily target their system [16].

Additionally, steroids have an impact on the tarsus, badge, wing bar, size, and beak. Size, color, wings bar, crest, and visual ability of the birds are all impacted by corticosterone [17]. Regardless of dose, the CORT-administered zebra finches had fewer copulations than the control animals. As a result, pair bonds are not significantly affected by acute CORT [18]. The effects of steroids on gender, sexuality, and the immune system in general. In females, humans, and animals, steroids increase illness and the immunological response. The most important finding is that gender and sex hormones have an effect on both the innate and the adaptive immune cells, but the mechanism responsible for this effect is unknown [5]. Recent research has demonstrated that 11beta-HSD serves both physiologic and pathological functions in the skin. In the context of the skin, the functions of 11beta-HSD include cell proliferation, the healing of wounds, inflammation, and the ageing process [19]. The goal of the current study was to explore the effects of steroids on the tissues of organisms as well as the pharmacotherapeutics and pharmaco-histokinetics of Bromocriptine as mesylate and estradiol valerate. This was accomplished through comparing the effects of Bromocriptine as mesylate and estradiol valerate on the serum and blood biochemistry of common quails that had either been subacutely or chronically stimulated with. The information was contrasted with that obtained for intact or control groups.

## 2. Materials and Methods

### 2.1. Ethical Approval

Institutional ethical approval for this study was obtained from the Ethical Committee of the Ghazi University, D G Khan, Punjab, Pakistan.

### 2.2. Experimental Birds

A total of 100 common quails are used during experimental periods (*Coturnix coturnix*). All of the birds are typically adult, weighing between 40 g and 150 g. These chickens are bought from D G Khan in a Pakistani chowk. The feed was manufactured at home without the use of medications and had sufficient nutrients (bajra, corn, and rice). Before beginning the treatment, all the birds had a five-day conditioning and adjustment period to the bird's condition.

### 2.3. Drug Formulation

Two medications were utilised over the course of the experiment. Each day, a brand-new Brotin and Pregnova solution is made and administered orally to all the birds receiving medication. The weight of the bird was used to calculate the required dosage of the medication formulation.

The article "The Comparative Pharmaco- and Histokinetics of the Therapeutic Dose of Estradiol Valerate and Bromocriptine in Common Quails" was retracted in 2024. Reasons: signs of a paper mill; suspected computer-generated content; unreliable results or conclusions; concerns about the data.

### 2.4. Dose Fixation

The dosage that was prescribed was the same as what was administered to the tiny mammals. The therapeutic dose is 2.5 mg/kg, and it is used to evaluate all of the potentially harmful effects of the whole medicine.

### 2.5. Therapeutic Dose

By using a syringe and a few tiny drops of steroid medication, the birds are administered their therapeutic dose.

### 2.6. Experimental Design

In each experiment, there were a total of 100 common quail birds, which were randomly divided into two groups of 50 birds each (summer and winter). In each experiment, there were a total of fifty birds, which were randomly assigned to one of three groups. Twenty birds were sacrificed in order to extract Brotin for drug testing. Twenty birds were sacrificed in order to collect Pregnova-treated medication samples. The remaining ten birds are split in half; five of them are utilised for the observation of clinical symptoms, while the other five are used to measure the treated birds' weights for comparison. The twenty birds are separated into four groups, each of which has five birds to make up its membership. Every trial lasts for a total of twenty days. Only five days of treatment were given to those five birds. The second group of five birds received treatment for somewhere between 1 and 10 days. The duration of treatment for the third group ranged from one to fifteen days. The duration of treatment for the fourth group ranges from 1 to 20 days. During the course of the experiment, each of the birds became completely accustomed to the setting in which they were placed. In order to reduce the amount of stress the birds were put through, it was necessary to take their rectal temperature and record their live body weight every five days. The birds' body weight was recorded in group 1, between 1 and 5 days. Between 1 and 10 days, group 2's total body weight is recorded every day. From day 1 to day 15, group 3 members had their body weight recorded. The participants in group 4 had their body weight recorded anywhere from 1 to 20 days. It has also been observed that the birds' temperatures are identical.

### 2.7. Clinical and Behavioral Observation

The birds were provided with fresh water and food three times a day, and their behavior and clinical status were monitored throughout the day. The behavioral observations made included the consumption of feed, dropping of the head, unrest, jumping in cages, and a feeling of hunger. Additionally, he was observed avoiding the other cage in order to hide in it.

The article "The Comparative Pharmaco- and Histokinetics of the Therapeutic Dose of Estradiol Valerate and Bromocriptine in Common Quails" was retracted in 2024. Reasons: signs of a paper mill; suspected computer-generated content; unreliable results or conclusions; concerns about the data.

### 2.8. Sample Collection and Processing

All of the birds in group 1 were given a thorough necropsy after 1 to 5 days, birds in group 2 were examined after 1 to 10 days, birds in group 3 were examined after 1 to 15 days, and birds in group 4 were examined after 1 to 20 days. In the event that there was a pathological alteration, this information is also documented. The sample was obtained from the kidneys, liver, and heart in addition to the skeletal muscles. For the purpose of histological analysis, representative tissue specimens were preserved in formalin at a concentration of 10%. Standard paraffin processing was utilised in order to preserve and embed the tissue. A section with a thickness of 5-6 m was cut. Eosin and hematoxylin were then used to stain the slides that had previously been prepared.

### 2.9. Histopathology Grassing

A location in the laboratory where the organ is sectioned off into parts measuring one centimetre in size. When the organ fragments are more than 1 centimetre in size, the reagent does not penetrate the tissue as well. The width of the samples is 1 centimetre, while the length is 1 inch. The ability to observe everything in the specimens, including colors, figures, and tumours, is one of the benefits of using this method. Following the cutting, fragments of the organs are placed in tissue cassettes and given labels before being stored.

### 2.10. Tissue Fixation

There are various fixatives employed, including ethylene, picric acid, and formaldehyde. Formaldehyde is utilised quite frequently in this context as a fixative. Formaldehyde can be purchased for a low price and is readily available in most marketplaces. Additionally, advantageous is the fact that it is readily absorbed by specimens. A formaldehyde solution is created through the process of diluting 37 percent of concentrated formaldehyde with 63 percent of water. This is done in accordance with the technique. After this step, take ten percent of it, combine it with ninety percent water, and utilise it in the fixation process. Formaldehyde should be left in contact with the tissue for a period of at least two hours and no more than sixteen.

### 2.11. Cutting Microtome

In cutting the tissue, a machine is used called a microtome. Different types of microtome are used, but here, a rotary microtome is used. This microtome is heavy and is fixed in place due to its weight. Parts are that holder which holds the tissue. The other is the cutter, where knives are used for cutting. Another part is the wheel which helps in cutting. After cutting the section, put it in hot water with temperature 50° to 60°C.

The article "The Comparative Pharmaco- and Histokinetics of the Therapeutic Dose of Estradiol Valerate and Bromocriptine in Common Quails" was retracted in 2024. Reasons: signs of a paper mill; suspected computer-generated content; unreliable results or conclusions; concerns about the data.

### 2.12. Staining

After removing the paraffin wax from the tissues, it was then immersed for three minutes in xylene. After that, the tissues are dipped into 100 percent alcohol for three minutes so that the xylene can be removed. The tissues are subjected to alcohol at concentrations ranging from 95 percent to 30 percent for a period of two minutes. In the five minutes that follow the alcohol, the tissues are soaked in water. For decolorization, a series of four to ten dips are performed, each using an ever higher grade of alcohol. In the subsequent 1 minute and a half to 2 minutes, eosin will be employed. The picture was then cleaned using xylene after three minutes of dehydrating the tissue to eliminate the alcohol. On the slide, a single drop of balsam from Canada was placed. On the slide, a cover slip was added before being fixed firmly.

## 3. Results

During the course of the trial, the clinical indications of somnolence and blindness of the eye with excessively dark speckled hues were detected in birds that had been treated with Pregnova. In the group that had been treated with Brotin, there were a few instances of diarrhoea that was bloody.

After 15 to 20 days of treatment, all clinical indications were observed in the groups who had been given medications. In comparison to the group that served as the control, the physiology of the birds' hearts and heart muscles showed no discernible signs of change (Figures 1 and 2). On the other hand, the drug-treated group's liver, kidneys, skeletal muscles, and heart showed little to no evidence of alteration. The micrographic picture of the heart in common quails during the first five days of treatment with Brotin, displays the congestion and hemorrhaging in tissues (Figure 3). When common quails were treated with Brotin in a ten-day trial, it displayed necrosis and inflammation in the heart's tissues and blood clotting in some heart tissues (Figure 4). The fifteen-day trial's common quails given Brotin displays inflamed fibroblasts and cardiac tissues (Figure 5).

The picture of the heart in common quails following a 20-day treatment with Brotin. It displays microhemorrhages and cardiac tissue irritation (Figure 6). Pregnova-treated common quail muscles in the first five days of a winter trial are depicted in a photo, with the muscles' unique areas of inflammation and fibroblast activity (Figures 7 and 8). Common quail's muscles in a photo representation from a ten-day winter study using Pregnova demonstrate the necrosis at certain muscle sites and fibroblast (Figures 9 and 10). Common quail muscles treated with Pregnova in a ten-day winter trial are depicted in a photo, with the muscles congested at certain locations and the vessels dilated (Figures 9 and 10). Common quail liver slices were photographed under a microscope to reveal typical histological features and characteristics (Figures 11 and 12). Common quail liver from a ten-day winter study with the drug Brotin is shown in the photo, with exudation at certain liver locations and significant hemorrhage (Figure 13). Photo representation of the common quail kidney after five days of Pregnova treatment, demonstrating inflammation and hemorrhages Figure 14). Common quail kidney was treated with Pregnova during a ten-day summer study, showing inflammation and hemorrhages (Figure 15). Common quail kidney was treated with Pregnova in a fifteen-day summer study, and the common quail kidney was treated with a photo representation of blood clotting and blood vessel break (Figure 16). Common quail kidney was treated with Brotin in a summer study for 20 days, displaying inflammation and inflammatory excaudate (Figure 17).

The article "The Comparative Pharmaco- and Histokinetics of the Therapeutic Dose of Estradiol Valerate and Bromocriptine in Common Quails" was retracted in 2024. Reasons: signs of a paper mill; suspected computer-generated content; unreliable results or conclusions; concerns about the data.

## 4. Discussion

The purpose of the current study was to investigate the effect that steroids have on the histopathology of common quail. In order to accomplish this goal, data were gathered through the conduct of experiments on common quail. In this chapter, we addressed the findings of the most recent study, which followed the empirical research that had been done previously on the histopathology of common quail. To begin, we will talk about the histological changes that have taken place in the tissues that are the focus of our investigation. Throughout the course of the trial with the common quail, a variety of clinical symptoms were noticed. These symptoms included a drooping of the head, an increase in hunger, hemorrhaging in the liver, body inflammation, and enteritis. The administration rate of steroids was found to be 27.0 percent in obese individuals, while it was only 11.9 percent in nonobese individuals. There was a significant disparity between the number of people who were fat and those who were not obese who used corticosteroids. It was shown that consuming corticosteroids causes a 10.5 percent rise in a person's body weight when they are already obese [13].

During the winter study, the birds that had been treated with Brotin displayed clinical signs of inflammation, including necrosis and a blood clot in the heart muscles. Throughout the course of the experiment, birds exhibit a variety of behaviors. Over the course of the test period of 10 days, there was a marginal shift in the weight of the birds. The weight of the birds in the experiment that were given Pregnova was found to be reduced, whilst the weight of the birds that were given Brotin was found to be increased. After 15 days of observation, each of the birds exhibited a distinct pattern of behavior in reference to their body weight. The experiment lasts for fifteen days, and at the end of that time, all of the birds have gained weight. The overall rise in the body weight of the birds was observed across all groups, including the control group as well as the experimental groups that received either Bromocriptine as mesylate or Pregnova. The clinical symptoms of kidney congestion, hemorrhages, and inflammatory excaudate were observed in the birds that had been treated with Brotin.

The article "The Comparative Pharmaco- and Histokinetics of the Therapeutic Dose of Estradiol Valerate and Bromocriptine in Common Quails" was retracted in 2024. Reasons: signs of a paper mill; suspected computer-generated content; unreliable results or conclusions; concerns about the data.

The weight of all of the different types of birds has increased. During this experiment, there was a significant shift in both the birds' outward appearance and their physical behavior. Some bird species get a dark area on their eye that appears to be tumours, and their skin develops a rough texture. There was a discernible change in the belligerent behavior of each and every bird. They are clearly agitated throughout the feeding procedures, and they attempt to break free from their stainless steel cages by making loud noises and squeezing the wire on the cages in an aggressive manner. Additionally, compared to the initial five to fifteen days of the trial, their hunger significantly increased.

Two weeks at a dose of 2 mg/kg/day, four weeks at a dose of 1 mg/kg/day, and three weeks at a dose of 0.4 mg/kg/day. The change was not particularly dramatic and did not represent a considerable departure from the baseline values. They exhibit some traces of impact despite the little amount of prednisolone that they took. The use of corticosteroids leads to an increase in mast cell degranulation as well as their production. Inhaled corticosteroids have also been demonstrated to induce inflammation, whereas the effects of corticosteroids mixed with those of beta-agonists have been shown to reduce the amount of inflammatory and allergic cell infiltration [20].

In the second experiment, which took place during the summertime, the actual weight of the birds exhibited varied patterns as a function of the food that they were given. During the course of the experiment, the birds' weight behavior consistently increased. When compared to Pregnova, the use of the steroid Bromocriptine as mesylate resulted in an increase in body weight that was more pronounced. During this test that lasted for 10 days, the conduct of the birds was astonishing in reference to their weight. Because we are using two separate steroids, each of these two steroids will have a unique effect. The birds that were fed Bromocriptine as mesylate consistently increased their weight, and they raised their weight day by day in comparison to the experiment that lasted five days.

The article "The Comparative Pharmaco- and Histokinetics of the Therapeutic Dose of Estradiol Valerate and Bromocriptine in Common Quails" was retracted in 2024. Reasons: signs of a paper mill; suspected computer-generated content; unreliable results or conclusions; concerns about the data.

The birds that were given with Brotin over the summer showed clinical symptoms of fibroblast, inflammation, and congestion. Both the winter and summer drug trials indicated relatively little changes in the organs; during the first five days of the Pregnova study, the participants gained weight; but, during the 10-day trial, they gradually lost weight. In this experiment, the birds behave less aggressively, but their medical examinations reveal that they have malignancies on the sides of their eyes. During the twenty-day winter trials of Brotin-treated birds, baldness was detected; however, during the twenty-day summer trials, baldness decrease occurred. After being observed for fifteen days, the birds behave in an unpredictable manner. The body weight of the birds that were treated with Bromocriptine mesylate saw an increase, while the body weight of the birds that were treated with Pregnova exhibited a reduction. The birds that were assigned to the control group saw a rise in their overall body mass. All three of these groups exhibited aggressive behavior [21], one as the control group and the other two as experimental groups.

During the summer study, birds that had been treated with Pregnova showed clinical indications consisting of modest dilatation of their kidney cells. There is a correlation between the size of a bird's body and its temperature. Because steroids alter the internal environment, this temperature varies erratically for no apparent reason. In addition to that, the temperature in the environment is quite hot during the summer months. During the summer trial, I discovered that the temperatures of the birds fluctuated when I administered steroid medications with brand names like Bromocriptine as mesylate and Pregnova. Every species of bird raises their body temperature, but to varying degrees. In general, the behaviors of birds were slightly altered, as evidenced by the fact that they displayed aggressive behavior, head-dropping inflammation, and particular patches on their legs. Also, birds will scratch their legs by pinching their beaks, which causes the scratching behavior. By inserting the thermometer into the anal region, the entire temperature was able to be determined with the assistance of a thermometer. A comparison of the tested member's liver with the livers of untested groups uncovered the fact that the tested member's liver displays a greater degree of change. In the course of the experimental investigation, steroids were utilised that had a considerable impact on their homeostatic function. The enzymes that are found in birds display a response to these steroids, which can also have an effect on the temperature of the birds. The temperature of the birds that were given Bromocriptine as mesylate constantly increased, and throughout the course of the trial's five days, the birds' temperature gradually declined [21].

The article "The Comparative Pharmaco- and Histokinetics of the Therapeutic Dose of Estradiol Valerate and Bromocriptine in Common Quails" was retracted in 2024. Reasons: signs of a paper mill; suspected computer-generated content; unreliable results or conclusions; concerns about the data.

The total effect of steroids on the temperature of birds was investigated over the course of twenty days, and during that time, the temperature did not change. There was not any discernible change in the temperature of the birds that were observed. Ovariectomized rats were used in this study to evaluate the effects of estradiol on the thermoregulatory responses brought on by methanol. For a period of two hours, the temperature was 270 or 160. When the temperature of the tail and the skin was taken at this point, it was found that the group that had been treated with methanol had a higher temperature than the rats that had not been treated with methanol. Because of this, the utilisation of methanol, which is a steroid, results in an increase in temperature [21].

The cumulative effect of consuming these steroids led to very unique and distinct manifestations of behavior. All of the birds exhibit very aggressive behaviors and vocalisations; they each pop their voices at different intervals and in varied ways. Steroids that are anabolic and androgenic are used to increase desire in both males and females for the purpose of sexual activity. Both relieving and contributing to depression are anabolic androgenic drugs. Increasing one's testosterone level might lead to aggressive behavior as well as psychological symptoms. Some anabolic steroids are generated synthetically, and the effects of taking them might lead to hypomania. Reduced steroid usage is another factor that contributes to depression [22].

Birds had a wide variety of other characteristics as well, the most notable of which was their tendency to sleep. According to the findings of that review, the effects of steroids on social interaction and neonatal periods led to a reduction in the activity level of birds to some degree. The neonatal phase is critical for the development of the neurological system as well as the ability to interact socially. In mammals, the neonatal phases are influenced by steroid use. The neonatal phase is a particularly delicate time for all mammals. Steroids and neuropeptides (such as oxytocin, arginine, and vasopressin) influence how people connect with one another socially. Neuropeptides are known to have an effect on a wide range of behaviors, including aggression, sociosexual behavior, parental conduct, and response to stress. Altering the levels of this hormone can cause changes in the social behavior of mammals [14].

The article "The Comparative Pharmaco- and Histokinetics of the Therapeutic Dose of Estradiol Valerate and Bromocriptine in Common Quails" was retracted in 2024. Reasons: signs of a paper mill; suspected computer-generated content; unreliable results or conclusions; concerns about the data.

## 5. Conclusion

Both trials of the steroids showed the expected clinical symptoms and histological alterations, with all processed groups corresponding to varying degrees of intensity among the various drugs. Differences in pharmacokinetic potency and histological response between different steroids are uncovered in the present investigation. Pregnova exhibits less severe unfavorable histotoxic effects on birds than Brotin, according to the most recent studies.

## Figures and Tables

**Figure 1:** Dissections of common quail Pregnova-treated birds. The dissection of common quail treated with Pregnova is done to compare it with controlled groups, and morphological characters have been observed keenly.

**Figure 2:** Dissections of common quail Brotin-treated birds. The dissection of common quail treated with Brotin is done to compare it with controlled groups, and morphological characters have been observed deeply.

**Figure 3:** Five-day winter trial Brotin-treated heart. The photomicrographic representation of the heart in common quails treated with Brotin in the first five days of trial. It shows the congestion and hemorrhages in the tissues of the heart.

**Figure 4:** 10-day summer trial Pregnova-treated heart. The photomicrographic representation of the heart in common quails treated with Brotin in ten days' trial. It shows the inflammation in the tissues of the heart and necrosis with blood clotting at some points of the tissues of the heart.

**Figure 5:** 15-day winter trial Brotin-treated heart. The photomicrographic representation of the heart in common quails treated with Brotin in fifteen days' trials. It shows the inflammation in the tissues of the heart and fibroblasts.

**Figure 6:** 20-day winter trial Brotin-treated heart. The photomicrographic representation of the heart in common quails treated with Brotin in twenty days' trial. It shows the inflammation in the tissues of the heart and microhemorrhages.

**Figure 7:** Histology of common quail normal bird's muscles (40x). Photomicrographic representation of quail's muscle sections was observed.

**Figure 8:** Five-day winter trial Pregnova-treated muscles. Photo representation of muscles of common quails treated with Pregnova in the first five days of the winter trial showed inflammation at specific muscle and fibroblast points.

**Figure 9:** 10-day summer trial Brotin-treated muscles. Photo representation of muscles of common quails treated with Pregnova in ten days of summer trial showed necrosis at specific muscle and fibroblast points.

**Figure 10:** 20-day summer trial Brotin-treated muscles. Photo representation of muscles of common quails treated with Pregnova in ten days of summer trial showed congestion at specific muscle points and dilation in the vessel.

The article "The Comparative Pharmaco- and Histokinetics of the Therapeutic Dose of Estradiol Valerate and Bromocriptine in Common Quails" was retracted in 2024. Reasons: signs of a paper mill; suspected computer-generated content; unreliable results or conclusions; concerns about the data.

**Figure 11:** Histology of common quail normal liver (40x). Photomicrographic representation of liver sections in common quails that shows normal histological parameters and structures.

**Figure 12:** Five-day summer trial Pregnova-treated liver. Photomicrographic representation of liver sections in common quails that shows normal histological parameters and structures.

**Figure 13:** 10-day winter trial Brotin-treated liver. Photo representation of the liver of common quails treated with Brotin in ten days of winter trial showed exudation at specific liver points and severe hemorrhages.

**Figure 14:** Five-day summer trial Pregnova-treated kidney. Photo representation of the kidney of common quails treated with Pregnova in five days of summer trial showing inflammation and hemorrhages.

**Figure 15:** 10-day winter trial Brotin-treated kidney. Photo representation of the kidney of common quails treated with Pregnova in ten days of winter trial showing inflammation and hemorrhages.

**Figure 16:** 15-day summer trial Pregnova-treated kidney. Photo representation of the kidney of common quails treated with Pregnova in fifteen days of summer trial showing blood clotting and bursting of the blood vessel.

**Figure 17:** 20-day winter trial Brotin-treated kidney (40x). Photo representation of the kidney of common quails treated with Brotin in twenty days of winter trial showing inflammation and inflammatory exudate.

## Data Availability

Data are available on request.
